# Totally thoracoscopic repair of atrial septal defect reduces systemic inflammatory reaction and myocardial damage in initial patients

**DOI:** 10.1186/2047-783X-19-13

**Published:** 2014-03-11

**Authors:** Xiang Liu, Yanhu Wu, Jinfu Zhu, Xiaoxia Lv, Yihu Tang, Jie Sun, Shijiang Zhang

**Affiliations:** 1 Department of Cardiothoracic Surgery, First Affiliated Hospital of Nanjing Medical University, Nanjing, China; 2 Department of Cardiothoracic Anesthesiology, First Affiliated Hospital of Nanjing Medical University, Nanjing, China

**Keywords:** Total thoracoscopy, Atrial septal defect, Cardiac surgery, Systemic inflammatory response, Myocardial damage

## Abstract

**Background:**

To compare the effect of totally thoracoscopic with conventional, open repair of atrial septal defect.

**Methods:**

Forty atrial septal defect cases were divided into two groups by surgical approach: totally thoracoscopic approach (group A, n = 20) and conventional open approach (group B, n = 20). In group A, surgical procedures were performed through three portal incisions in the right lateral chest wall under thoracoscopic vision without the aid of a computerized robotic surgical system. Notably, all operations were completed by one surgeon who had just begun using this technique. In group B, the atrial septal defects were repaired in conventional open fashion. Clinical outcomes and serum levels of tumor necrosis factor α (TNF-α), interleukin-6 (IL-6), interleukin-10 (IL-10), intercellular adhesion molecule 1 (ICAM-1), and creatine kinase isoenzyme-myocardial band (CK-MB) for the two groups were evaluated and compared.

**Results:**

All operations were performed successfully without serious complications. Durations of cardiopulmonary bypass (CPB), CPB setup, aortic cross-clamping, and operative procedure were significantly longer in group A than in group B (*P* < 0.05). The recovery times for body temperature and laboratory values of leukocytes were significantly shorter for group A than for group B (*P* < 0.05). There were no differences in durations of postoperative assisted ventilation or intensive care unit and hospital stays, volumes of blood transfused intraoperatively or thoracic drainage, or medical costs between the two groups. Serum levels of inflammatory factors (TNF-α, IL-6, IL-10, and ICAM-1) and CK-MB increased significantly in both groups after surgery. However, 6 h and 12 h after surgery, levels of these inflammatory factors and CK-MB were significantly lower in group A than in group B (*P* < 0.05).

**Conclusions:**

Thoracoscopic cardiac surgery is technically feasible and safe, with less trauma and quicker recovery even when done by a surgeon newly introduced to the technique.

## Background

Repair of atrial septal defect (ASD) using a totally thoracoscopic approach is the oldest and most popular application of video-assisted thoracoscopic cardiac surgery [1-3]. Since 2008, we have carried out ASD repair using a totally thoracoscopic approach with satisfactory clinic results and without the aid of a computerized robotic surgical system. However, thoracoscopic cardiac surgery is still controversial because its minimally invasive nature makes the surgery longer and more difficult, especially because of the newness of this technique. In the present study, to evaluate the advantages of this method when performed by a surgeon newly introduced to this technique, we compared the outcomes of thoracoscopic cardiac surgery in 20 consecutive patients with those of conventional thoracotomy with regard to postoperative systemic inflammatory response syndrome (SIRS) and myocardial injury.

## Methods

### Patients and surgeon

Forty patients from our hospital who were diagnosed with ASD and underwent repair between 2010 and 2012 were divided into two groups: totally thoracoscopic (group A, n = 20) and conventional open (group B, n = 20) surgical approaches. Echocardiograms demonstrated ASD without other cardiovascular anomalies. Only patients who could not undergo percutaneous interventional closure because of defect size or ASD type were included. Various factors including age, sex, weight, cardiothoracic ratio, cardiac function as demonstrated by ejection fraction, size of ASD, and hematocrit were compared. There were no significant differences in these parameters between groups (Table 1). Both methods were considered feasible in the hospital. Patient consent was not deemed necessary by the local research and ethics committee (Nanjing Medical University Institutional Review Board).

**Table 1:** Patient baseline characteristics

	**Group A**	**Group B**	***P *** **value**
**Variables**	**(n = 20)**	**(n = 20)**	
Age (years, mean ± 1SD)	22.13 ± 2.2	27.95 ± 2.3	0.073
Gender (male)	9 (45%)	6 (30%)	0.327
Weight (kg, mean ± 1 SD)	51.13 ± 12.2	51.43 ± 8.8	0.932
Cardiothoracic ratio (%, mean ± 1 SD)	52 ± 4.9	53.55 ± 3.6	0.281
EF (%, mean ± 1 SD)	65.53 ± 4.1	68.61 ± 5.2	0.067
Size of ASD (mm, mean ± 1 SD)	29.87 ± 4.73	26.83 ± 7.42	0.182
Hematocrit (%, mean ± 1 SD)	0.39 ± 0.04	0.39 ± 0.03	0.816

*ASD*, atrial septal defect; *EF*, ejection fraction; *SD*, standard deviation.

Thoracoscopic cardiac surgeries were performed by one surgeon newly introduced to this technique. The surgeon’s preoperative preparation included attaining a large amount of theoretical knowledge of endoscopy and carrying out a great deal of endoscopic, especially thoracoscopic, training; mastery of routine and minimally invasive cardiac surgeries and demonstrating the ability to deal with unexpected situations independently; mastery of thoracic surgical skill and ability to be trained in total thoracoscopic lung lobectomy; practice performing the techniques on pigs; and observation of totally thoracoscopic cardiac surgery at other hospitals.

### ASD surgical repair

The patients in group A were placed under endotracheal anesthesia via a double-lumen endotracheal tube and the femoral artery and vein were cannulated. Left single-lung ventilation was applied. Oxygen saturation was monitored. If oxygen saturation fell below 90%, double-lung ventilation was initiated. A 2-cm-long incision was made in the fifth intercostal space at the right midaxillary line. A trocar was placed through the incision and the thoracoscope (Stryker Inc., Kalamazoo, MI, USA) was inserted through the trocar. Another 2-cm incision was made parasternally at the third intercostal space for insertion of surgical instruments and the inferior vena cava snare. A third 2-cm incision was made in the second intercostal space at the right mid-axillary line for insertion of surgical instruments, the superior vena cava snare, a cannula for cold perfusion, and an aortic clamp (Figure 1). For all intrathoracic procedures, the surgical field was displayed on a screen and a computerized robotic surgical system was not employed. The ASD was closed with direct running suture and in some cases reinforced with a Dacron patch. Group B patients underwent with single-lumen endotracheal anesthesia and conventional cardiopulmonary bypass (CPB). Patients were positioned supine for access to the mid-sternal surgical area.

**Figure 1:** Surgical incisions and portal sites.

All patients were anesthetized using fentanyl 10-20 μg/kg, midazolam 0.1-0.15 mg/kg, isoflurane 0.2-1.5%, and/or propofol 50-100 μg/kg/min. Muscle relaxation was achieved with rocuronium 0.6-1.0 mg/kg. Heparin was given to maintain an activated clotting time (ACT) >420 s during CPB. Bypass management included membrane oxygenation (Affinity NT; Medtronic Inc., Fridley, MN, USA) and maintenance of mean arterial pressure between 55 and 85 mmHg, temperature between 32 and 35°C, and blood sugar between 4 and 10 mmol/L. Myocardial protection was achieved with cold blood crystalloid cardioplegia, and terminal warm-blood cardioplegic reperfusion (a hot-shot) of 250-500 mL was delivered just prior to the removal of the aortic cross-clamp. After the patient came off CPB, heparin was reversed with protamine (approximately 10 mg/1,000 units of heparin). Postoperatively, patients were managed in a specialized cardiovascular intensive care unit with standardized protocols for early extubation and blood glucose control (target 5.1 to 8.0 mmol/L).

### Clinical outcome measures

Volumes of blood transfused and thoracic drainage; durations of CPB setup, CPB, aortic cross-clamping, the operative procedure, postoperative assisted ventilation, and ICU and hospital stays; and medical costs were recorded for both groups.

### Blood sampling and measurement

Whole venous blood (10 mL) was taken from all patients preoperatively; immediately after aortic opening; and 2, 6, 12, 24, and 72 h postoperatively. The samples were centrifuged for 10 min at 3,200 rpm, and the supernatants were collected and preserved at -80°C. Levels of tumor necrosis factor-α (TNF-α), interleukin-6 (IL-6), intercellular adhesion molecule-1 (ICAM-1), interleukin-10 (IL-10), and creatine kinase isoenzyme-myocardial band (CK-MB) were measured by enzyme-linked immunosorbent assay (ELISA) using commercially available ELISA kits (ADL Biotech Inc., Mashteuiatsh, QC, Canada). All tests on samples and standards were performed in duplicate per manufacturer instructions.

### Statistical analysis

Statistical analysis was performed using SPSS for Windows, Version 13.0 (SPSS Inc., Chicago, IL, USA). All variables are presented as mean ± standard deviation (SD). Patient baseline characteristics (except sex, which was compared using the *χ*^2^ test) and operative results were compared with independent *t*-tests. One-way analysis of variance was used to analyze serum levels of inflammatory factors and CK-MB. A value of *P* < 0.05 was considered statistically significant.

## Results

All operations were performed successfully without serious complications. Patients in both groups were cured and were followed for a mean of 24 months (range, 18 to 34 months). All patients could return to work and activities of daily living and had no long-term complications.

The recovery times for body temperature and laboratory values of leukocytes were significantly shorter for group A than for group B (Table 2). There were no differences between the two groups in durations of postoperative assisted ventilation or ICU and hospital stays; no differences in volumes of blood transfused or thoracic drainage, and no difference in medical costs (Table 2). Durations of CPB, CPB setup, ascending aortic cross-clamping, and operation were significantly longer in group A than in group B (Table 2).

**Table 2:** Operative results

	**Group A**	**Group B**	***P *** **value**
**Variables (mean ± 1 SD)**	**(n = 20)**	**(n = 20)**	
CPB time (min)	82.75 ± 18.8	52.45 ± 9.9	<0.001
CPB setup time (min)	88.44 ± 17.13	52.05 ± 21.00	<0.001
Aortic cross-clamping time (min)	44.31 ± 12.9	25.31 ± 11.8	0.002
Operation time (h)	4.92 ± 0.7	3.31 ± 0.7	<0.001
Recovery time for body temperature (d)	3.13 ± 2.10	5.68 ± 5.20	0.036
Recovery time for laboratory values of leukocytes (d)	4.31 ± 2.20	7.96 ± 5.00	0.003
Postoperative respirator-assisting time (h)	13.63 ± 7.92	11.15 ± 5.87	0.289
Units of erythrocytes transfused (U)	3.4 ± 1.9	3.0 ± 1.8	0.477
Amounts of plasma transfused (mL)	753.1 ± 462.8	685.0 ± 291.1	0.593
Thoracic drainage volume (mL)	327.8 ± 219.7	288.5 ± 182.1	0.561
Length of ICU stay (h)	20.9 ± 8.6	21.7 ± 7.7	0.78
Length of hospital stay (days)	10.38 ± 1.36	12.30 ± 4.80	0.102
Medical cost (Ұ,RMB)	42,637 ± 4,774.3	39,546 ± 7,974.8	0.181

*CPB*, cardiopulmonary bypass; *ICU*, intensive care unit; *RMB*, Renminbi (Chinese currency); *SD*, standard deviation.

Serum levels of inflammatory factors (TNF-α, IL-6, ICAM-1, IL-10) and CK-MB did not differ significantly between groups before CPB but significantly increased after CPB.

TNF-α levels peaked 6 h after aortic opening in both groups. Values for group B were higher than those for group A at each time point of CPB and differed significantly at 0 h (immediately after aortic opening) and 6, 12, and 24 h after aortic opening (Figure 2).

**Figure 2:** **Expression of TNF-α in groups A and B.** *P < 0.05.

IL-6 levels peaked 6 h after aortic opening in both groups. Group B IL-6 values were greater than those for group A at each time point of CPB and differed significantly at 2 and 12 h after aortic opening (Figure 3).

**Figure 3:** **Expression of IL-6 in groups A and B.** *P < 0.05.

Levels of ICAM-1 peaked 2 h after aortic opening in both groups. ICAM-1 values were greater in group B than in group A at each CPB time point and were significantly different at 2, 6, and 24 h after aortic opening (Figure 4).

**Figure 4:** **Expression of ICAM-1 in groups A and B.** *P < 0.05.

IL-10 levels of IL-10 peaked 12 h after aortic opening in both groups, with a value significantly higher in group B than in group A 12 h after aortic opening (Figure 5).

**Figure 5:** **Expression of IL-10 in groups A and B.** *P < 0.05.

CK-MB level peaked 6 h after aortic opening in group A and 24 h after aortic opening in group B, with values greater in group B than in group A at each CPB time point and significant differences seen 6, 24, and 72 h after aortic opening (Figure 6).

**Figure 6:** **Expression of CK-MB in groups A and B.** *P < 0.05.

## Discussion

One of the current arguments against totally thoracoscopic cardiac surgery is that it does not comply with the requirements of minimal invasion because the durations of CPB and ascending aortic cross-clamping associated with this method are significantly prolonged [4-6]. Open ASD repair is usually completed by a junior surgeon, and a senior surgeon often acts as instructor and assistant. Therefore, operative duration, including CPB and aortic cross-clamping, were longer in group B. Nevertheless, durations of CPB, CPB setup, aortic cross-clamping, and operation in group B were significantly shorter than in group A. The corresponding activation of SIRS after CPB in group A should be more serious and may cause severe impairment of organ function; thus, because of potential trauma to the patient, the thoracoscopic technique does not meet the claim of minimal invasion. Especially since this work had just begun, durations of CPB, CPB setup, ascending aortic cross-clamping, and operation in group A were not only significantly longer than in group B, but also longer than in thoracoscopic cardiac surgical procedures completed by a skilled and experienced doctor [3,7].

SIRS occurs after CPB mainly because of the contact of blood with foreign body surfaces during CPB. This leads to multi-system and multi-cell activation and produces a large number of humoral and cellular inflammatory mediators through a cascade reaction, which eventually causes tissue and organ damage or even multiple organ dysfunction syndrome [8-10]. Causes of SIRS also include surgical injury, anesthesia, changes in body temperature, organ ischemia/reperfusion injury, machine blood transfusion, hemodilution, and heparin-protamine complexes [11,12]. It is important to understand the claim of minimal invasion of totally thoracoscopic cardiac surgery apart from the size of the incision.

Levels of TNF-α, IL-6, and ICAM-1, which are the main inflammatory cytokines occurring after CPB and which play critical roles in the inflammatory cascade, are important in evaluating SIRS after CPB. They are released first and are also the most important endogenous mediators in the inflammatory process after CPB [13-15]. In the present study, we found that in patients who underwent totally thoracoscopicASD repair, levels of TNF-α, IL-6, and ICAM-1 increased early on and were significantly higher than the increased values induced by CPB, aortic cross-clamping, and other operation. However, in patients who underwent thoracoscopicASD repair, elevations in the levels of TNF-α, IL-6, and ICAM-1 were of short duration, dropped soon after operation, and were significantly lower than those in patients who underwent open surgery at the same period. Our finding suggests that the degree of SIRS activated by totally thoracoscopicASD repair is lower than that in conventional surgery if other factors, such as recovery from surgical trauma and postoperative cardiopulmonary function, are included.

The prognosis of SIRS after CPB also depends on another important factor, the balance between proinflammatory factors and anti-inflammatory factors. IL-10 is an important post-CPB anti-inflammatory factor that has an endogenous protective effect that counters tissue and cell destruction caused by inflammatory mediators [15,16]. However, if the anti-inflammatory response to SIRS is too strong, it will reduce immune function and increase the body’s susceptibility to infection, and induce or aggravate multiple organ failure. The compensatory anti-inflammatory response syndrome (CARS) is a complex pattern of immunologic responses to severe infection or injury. Many studies have shown that the timing and relative magnitude of these responses have a profound impact on patients’ outcomes [17,18]. Our study suggests that the level of the anti-inflammatory cytokine IL-10 in totally thoracoscopicASD repair maintains good homeostasis with levels of inflammatory cytokines, reaches a peak in the early postoperative period, and drops quickly. The peak value is also lower than that in conventional surgery, which indirectly reflects the smaller systemic inflammatory response of thoracoscopic cardiac surgery.

CK-MB level in serum increases when there is myocardial injury. It is widely used to determine perioperative myocardial injury after cardiac surgery and is an important indicator of the recovery of cardiac function and prognostic risk factors [19,20]. The present study has shown that the extent of myocardial injury after thoracoscopicASD repair was significantly lower than after conventional surgery, which is a prerequisite for the successful rehabilitation of patients who undergo cardiac surgery.

The main reasons for SIRS and myocardial injury are CPB and surgical injury. Compared with conventional thoracotomy, thoracoscopic cardiac surgery avoids a large chest incision and sternotomy wound, significantly reduces tissue damage, and maintains the overall structure of the thorax. In addition, the blunt trauma of endoscopic surgery, such as stretching and squeezing the heart, is greatly decreased. Thus, thoracoscopic cardiac surgery may prevent SIRS and myocardial injury.

## Conclusions

Although it is more difficult and dangerous, after careful preparation, thoracoscopic cardiac surgery is technically feasible and creates less trauma and quicker recovery. In addition, thoracoscopicASD repair, which can be characterized as minimally invasive, results in a reduced systemic inflammatory response after CPB, maintains the balance of proinflammatory and anti-inflammation factors, reduces tissue and organ damage, even when performed by a surgeon new to this technique.

## Abbreviations

ASD: Atrial septal defect; CARS: Compensatory anti-inflammatory response syndrome; CK-MB: Creatine kinase isoenzyme-myocardial band; CPB: Cardiopulmonary bypass; ELISA: Enzyme-linked immunosorbent assay; ICAM-1: Intercellular adhesion molecule-1; ICU: Intensive care unit; IL-6: Interleukin-6; IL-10: Interleukin-10; RMB: Renminbi (unit of Chinese currency); SD: Standard deviation; SIRS: Systemic inflammatory response syndrome; TNF-α: Tumor necrosis factor-α

## Competing interests

The authors declare that they have no competing interests.

## Authors’ contributions

YHW conceived and designed the experiments. XL analyzed the data and wrote the manuscript. XXL and YHT performed blood sampling and the experiments. SJZ supervised the study, participated in its design and coordination, and drafted the manuscript. JFZ and JS advised on clinical implications. All authors read and approved the final manuscript.
